The article "Highly dispersed silver imbedded into TiN submicrospheres for electrochemical detecting of hydrogen peroxide" was published in 2020. Journal: Sci Rep.

# Highly dispersed silver imbedded into TiN submicrospheres for electrochemical detecting of hydrogen peroxide

**DOI:** 10.1038/s41598-020-79286-y

**Published:** 2020-12-17

**Authors:** Youqun Chu, Zhangkao Huang, Xinhang Wang, Menglei Zhou, Fengming Zhao

**Affiliations:** State Key Laboratory Breeding Base of Green Chemistry-Synthesis Technology, College of Chemical Engineering, Zhejiang University of Technology, Hangzhou City, 310032 Zhejiang China

**Keywords:** Analytical chemistry, Electrochemistry, Electrocatalysis

## Abstract

We report the fabrication of silver nanoparticles evenly imbedded into TiN submicrospheres via one-pot solvothermal reaction and subsequent nitridation for electrochemical detecting of hydrogen peroxide. The precursor of TiO_2_ submicrospheres and high dispersion of silver nanoparticles are regulated by the alcoholysis of tetrabutyl titanate and reducibility of enol in vitamin C. The ion nitriding promoted the conductivity and micro-nano porous structure on the surface of TiN submicrospheres, which increase the dispersity of silver nanoparticles and make contributions to avoid aggregations. More importantly, the electrochemical response of Ag-TiN submicrospheres to H_2_O_2_ was remarkably enhanced due to the co-effects of Ag and N-doping. It provides a superior sensing performance for electrochemical detection of hydrogen peroxide at − 0.3 V with a high sensitivity of 33.25 μA mmol L^−1^ cm^−2^, wide linear range of 0.05–2100 μM and low detection limit of 7.7 nM. The fabricated sensor also reliably applied in detection of H_2_O_2_ in milk samples with good reproducibility, repeatability and storage stability.

## Introduction

Hydrogen peroxide (H_2_O_2_) plays crucial roles in chemical industries, clinical analysis and physiological process^1^. In biomedical systems, if the concentration of H_2_O_2_ exceeds the permissible limit (> 700 nM)^2^, it will be associated with diabetes, cardiovascular diseases, Alzheimer`s disease, cancer, and so on^3–5^. Rapid and accurate detection of H_2_O_2_ is beneficial to monitor the quality of human health and industrial processes^6^. Therefore, various analytical protocols have been reported for H_2_O_2_ assay, including chemiluminescence^7^, spectrometry^8^, fluorescence^9^ and electrochemistry sensors^10–12^. Among them, electrochemical technology, especially enzyme-free model^13^, has recently received more research interests due to its rapidity, economy and capability for in situ sensing H_2_O_2_. Up to now, a great deal of efforts have been devoted to the development of non-enzymatic electrochemical sensors based on silver nanoparticles^14^, which have been proven to be an inexpensive, nontoxic and highly effective catalyst for amperometric H_2_O_2_ detection^15^. However, agglomeration between silver nanoparticles because of strong van der Waals force always results in a sharp decrease of electrocatalytic activity and stability^16^. Thus, the urgent task is to create a convenient means for repeatable synthesis of finely dispersive silver with greater stability. This task is still of significant importance to construct a stable silver-based sensor for clinical analysis, biomedical systems and other fields, in which implying the long-term stability. Therefore, it is necessary to further develop a synthetic route to obtain aggregative stability of silver dispersions with improved electrochemical performance.

Many methods have been proposed for the preparation of highly dispersed silver, such as spray pyrolysis^17^, electrolysis^18^, microwave plasma^19^, and chemical liquid-phase reduction process^20^. Most of the reported literatures focused on controlling the size of silver, while little on the dispersibility and few on dispersive mechanism. Immobilization of silver on organic or inorganic scaffolds has been proved to be an effective strategy against agglomeration with the improved stability^21–23^. Nanostructured titanium oxides as important multi-valent compound, including TiO, Ti_2_O_3_ and TiO_2_, can be employed as the scaffold for silver due to their unique electrical property, non-toxic, and chemical stability. Furthermore, titanium oxides have the characteristic of controllability in micro-scale construction, which provides an efficient way to load silver. However, changes in the crystalline phase, shape and conductivity of microstructure could have led to reliability at load that caused in the availability of carrier materials for sensors^24–26^. It has been reported that doping with nitrogen could enhance the interior conductivity of TiO_2_ due to the uniform distribution of dopants throughout the particles. As successful examples, a sugar-apple-like N-doped TiO_2_@ carbon core–shell spheres as high-rate and long-life anode materials has been synthesized by carburizing and nitriding, while the conductive N-doped carbon shell with slit pores uniformly coated on TiO_2_ spheres surface revealing superior long-term cycling stability for lithium ion batteries^27,28^. Furthermore, titanium nitride (TiN) has attracted extensive interests as carrier materials because of super high electrical conductivity, biocompatibility and chemical stability^29–31^. Biocompatible TiN nanorod arrays fabricated by solvent-thermal synthesis and subsequent nitridation in ammonia atmosphere deliver the superior electrocatalytic activity and highly selective sensing H_2_O_2_ owing to their good electronic conductivity and large surface area^32^. Robust TiN nanotubes supported Pt catalyst with enhanced catalytic activity and durability for methanol oxidation reaction exhibit small size, good dispersion and fast electron transfer due to the strong metal-support interactions of TiN nanotubes^33^. Recent researches show TiN can be employed in a wide range of applications such as biosensing^32^, pH-sensitive material^34^, electroanalysis^35^, supercapacitors^36^, and energy storage^37^. Therefore, TiN can better be employed as the scaffold for silver because of their high chemical and physical stability, environmentally non-toxic and unique electrical property. Furthermore, the electrocatalytic ability of TiN might promote the synergistic effects of silver highly dispersed nanocomposites for H_2_O_2_ sensors.

In the present work, nonstoichiometric single phase TiN was employed as scaffold and solvothermal pathways in harmoy of silver dispersion and subsequent nitridation using ammonia annealing. In the solvothermal process, vitamin C in ethanol was used as a reducing agent to get the silver evenly distributed in TiN submicrospheres. Figure 1 displays the synthesis procedure for fabrication of Ag-TiN submicrospheres. Benefiting from its inexpensive, simple synthetic route and extraordinary properties for H_2_O_2_ detection, this novel material is a hopeful candidate in the development of efficient nonenzymatic H_2_O_2_ sensor.

**Figure 1:** Scheme illustration of the synthesis procedure of fabrication of Ag-TiN submicroshperes for H_2_O_2_ sensor.

## Methods

### Materials and reagents

The materials and reagents for synthesizing Ag-TiN submicrospheres (Ag-TiN/SMS) are sliver nitrate (AgNO_3_, 99.8%), vitamin C (VC, 99.7%) and tetrabutyl titanate (TBOT, 99.0%) acquired from Aladdin, China. The reagents include hydrogen peroxide (H_2_O_2_, 30%), uric acid (UA, 99.0%), L-glucose (L-Glu, 98%), glycine (Gly, 99%) and lactosum (Lac, 98%) were acquired from Aladdin, China. Glassy carbon (GC, ϕ 3.0 mm) electrode was washed by deionized water. Phosphate buffer solution (PBS, pH = 7.0, 0.02 M) as supporting electrolyte was prepared with KH_2_PO_4_ and KOH (Sinopharm, China).

### One-step hydrothermal process of Ag-TiO_2_ submicrospheres (Ag-TiO_2_/SMS)^38^

In the paper, vitamin C (30 mmol) and AgNO_3_ (30 mg) were added to absolute ethanol (70 mL) with magnetic stirring, and then adding TBOT (8 mmol) to solution drop by drop form clear to brown color (Ag / Ti source (m %) is 10%). Subsequently, the mixture was transferred into 100 mL Teflon-line stainless autoclave (Microreactor, Yanzheng Instrument Ltd. Shanghai) and heated in the oven at 200 °C for 7 h. After cooled down in air, the solid product was separated by centrifugation, washed with deionized water and absolute alcohol several times, and dried in a vacuum at 60 °C for 6 h.

### Reduction and nitridation of Ag-TiN/SMS^39^

The precursor of Ag-TiO_2_/SMS was kept in a horizontal quartz furnace. A flow of N_2_ (99.999%) with a rate of 100 mL min^−1^ was introduced to remove air and moisture for 30 min. Then the furnace was heated from room temperature to 450 °C at a rate of 20 °C ⋅min^−1^ and the Ag-TiO_2_/SMS was annealed for 1 h. After the furnace temperature was sequentially heated from 450 °C to 850 °C, the flowing gas was switched to NH_3_ (160 mL min^−1^) and the nitriding reaction was carried out for 2 h. Finally, the Ag-TiN/SMS were cooled via purging nitrogen gas.

### Preparation and characterization of Ag-TiN/SMS electrode

GC (φ = 3.0 mm, S = 0.0707 cm^2^) was polished by aluminum oxide powders(300 nm and 50 nm respectively), and subsequently washed with acetone, ethanol and deionized water successively for several times. 2.0 mg Ag-TiN/SMS mixed with 100 μl deionized water, 100 μl absolute ethanol and 10 μl 5%Nafion as mixture, and the mixture was sonicated for 30 min. The Ag-TiN/SMS electrode for H_2_O_2_ detection were prepared as follows: 3.5 μl the mixture was dropped on the surface of GCE and waited to dry in ambient air.

The morphology of TiN/SMS and Ag-TiN/SMS were displayed by scanning electron microscope (SEM), high resolution transmission electron microscopy (HR-TEM) and high angle annular dark field scanning transmission electron microscopy (HAADF-STEM). In addition, analysis of chemical elements in materials was demonstrated by energy dispersive X-ray spectrometer (EDX), using Cu-Kα radiation and spherical-aberration corrected field-emission TEM (Philips-FEI, Tecnai G2 F30 S-Twin). The crystalline structure of TiN/SMS and Ag-TiN/SMS were analysed by X-ray diffractometer (XRD, PNAlytical),using Cu-Kα as X-ray source and scaning in the range of 20°–80°. The oxidation states of Ag-TiN/SMS were detected by X-ray photoelectron spectroscopy (XPS, Kratos Axis Ultra DLD) using a focused monochromatized Al-Kα operated at 300 W. The binding energies were referenced to the C1s line at 284.6 eV from adventitious carbon.

### Electrochemical property and amperometric response to H_2_O_2_

Electrochemical property measurements were demonstrated on Ivium potentiostat in 0.02 M PBS (pH 7.0) with different concentrations of H_2_O_2_.The detection of H_2_O_2_ by cyclic voltammetry using a three-electrode cell such as the Ag-TiN/SMS as working electrodes, Pt foil as counter electrode and Ag/AgCl as reference electrode. The electrochemical impedance spectroscopy (EIS) was detected by applying 5.0 mV amplitude at a frequency of 100 kHz to 10 MHz. In order to research the selectivity, long-term stability, reproducibility and repeatability of Ag-TiN/SMS. This paper adopted chronoamperometry to compare the response current. The chronoamperometry were also performed in 0.02 M PBS (3.0 mL, pH 7.0) at − 0.3 V. Real sample detection was attested by adding different concentrations of H_2_O_2_ solutions to the pre-treated milk sample (3.0 mL, pH 7.0).

## Results and discussion

### Characterization of Ag-TiN/SMS

Figure 2 shows a typical SEM image of the TiN/SMS (a), Ag-TiN/SMS (b) and TEM images of TiN/SMS (c–e), Ag-TiN/SMS (f–h). The surface of the sample is roughened by rupturing the layers of material surface after nitridation. Hierarchical Ag-TiN/SMS (b) have a higher surface roughness. Silver remains highly dispersed on the surface of TiN. The average diameter of the Ag-TiN/SMS is of 150–250 nm.

**Figure 2:** SEM images of TiN/SMS (**a**) and Ag-TiN/SMS (**b**); TEM images of TiN/SMS (**c**–**e**) and Ag-TiN/SMS (**f**–**h**).

The morphology and microstructure of TiN/SMS (a) and Ag-TiN/SMS (b) are further studies using high resolution transmission electron microscopy (HR-TEM). Figure 2 c,f show low-magnification TEM images, which reveal the detailed structure of the spherical morphology. TiN/SMS and Ag-TiN/SMS actually are composed of many individual nanoparticles, which may further give rise to a porous structure. Figure 2d,e show high-magnification TEM images of TiN/SMS. As shown In Fig. 2e, TiN/SMS have interplanar distances of 0.211 nm, which can be attributed to the TiN (200) plane. Figure 2g,h show high-magnification TEM images of Ag-TiN/SMS. Ag^0^ were grown on the surface of Ag-TiN/SMS. These NPs are highly crystalline and the lattice fringe presented in the high-resolution TEM image. In Fig. 2h, the interplanar distances of Ag-TiN/SMS was 0.211 nm and 0.236 nm, which can be attributed to the TiN (200) plane and Ag (111) plane.

Furthermore, EDX of TiN/SMS and Ag-TiN/SMS also have been investigated. The Fig. 3a illustrated that the Ti, O, N elements were included in the TiN/SMS, and the Fig. 3b shows final materials have N element except to Ti, O and Ag, indicating that titanium nitride can be obtained after nitriding. The distribution of N element is relatively homogenous in TiN/SMS (c) and Ag-TiN/SMS (d), which is proved by the corresponding elemental mapping images (Fig. 3c,d). Silver remains highly dispersed over the surface of the submicrospheres.

**Figure 3:** EDX Drift corrected spectrum images of TiN/SMS (**a**) and Ag-TiN/SMS (**b**); HAADF-STEM images and the corresponding EDX element mapping of TiN/SMS (**c**) and Ag-TiN/SMS (**d**).

Figure 4 is the P-XRD patterns of TiN/SMS and Ag-TiN/SMS. For TiN/SMS sample, the diffraction peaks appeared at 36.9°, 42.8°, 62.2°, 74.5° and 78.4° can be indexed as TiN (111), (200), (220), (311)and (222) crystal planes. Four peaks with a value of 2θ around 38.1°, 44.3°, 64.4° and 77.4° can be assigned to Ag (111), (200), (220) and (311) plants in Ag-TiN/SMS sample. However, the diffraction peak of silver is much stronger than that of titanium nitride. It may be related to the high dispersion of silver on the surface of titanium nitride.

**Figure 4:** P-XRD patterns of TiN/SMS and Ag-TiN/SMS.

Figure 5 shows the XPS high resolution spectrum of Ti 2p (a), O 1s (b), N 1s (c), Ag 3d (d) and Ag MVV (e) for Ag-TiN/SMS. Ti 2p spectra is complex and can be divided into Ti 2p_1/2_ and Ti 2p_3/2_ peaks. For Ti 2p_1/2_, the peaks at 459.9 eV, 461.4 eV and 463.2 eV can be assigned to Ti–N, Ti–N–O and Ti–O bonds, which are consistent with the literature. The binding energies of 454.7 eV, 456.0 eV and 457.7 eV are associated with Ti–N, Ti–N–O and Ti–O bonds, respectively. The N 1s region for Ag-TiN/SMS shows peaks at 395.4 eV, 396.4 eV and 400.8 eV that are commonly ascribed to Ti–N, Ti–N–O and N–C bonds. The O 1sregion for Ag-TiN/SMS shows peaks at 529.2 eV and 530.9 eV that are commonly ascribed to Ti–O and Ti–N–O bonds, respectively. The Ag3*d* core-level spectra of Ag-TiN/SMS exhibit well defined double peak formations located at binding energies of 368.0 eV and 374.0 eV, corresponding to the Ag3d_5/2_ and Ag3d_3/2_, respectively. The difference of about 6.0 eV between these two binding energies verifies the formation of Ag^0^ in Ag-TiN/SMS. As shown in the Ag MVV spectra, the peak appeared at 358.0 eV and the Auger parameters (α′) is calculated to be 726.0 eV, which is ascribed to Ag^0^ in Ag-TiN/SMS.

**Figure 5:** XPS spectra of Ag-TiN/SMS of (**a**) Ti 2p, (**b**) O 1s, (**c**) Ag 3d, (**d**) N 1s and (**e**) Ag MVV.

### Electrochemical performance of Ag-TiN/SMS

Figure 6 showed the cyclic voltammograms of TiN/SMS (a) and Ag-TiN/SMS (b) electrodes at the scan rate of 20 mV⋅s^−1^ with addition different concentrations of H_2_O_2_. Ag-TiN/SMS showed a prominent and enhanced reduction peak current at approximately − 0.45 V. This excellent electrocatalytic response to H_2_O_2_ is much higher than on the TiN/SMS at the same conditions, suggesting Ag-TiN/SMS had better reduction ability for H_2_O_2_ reduction. Moreover, this also demonstrates that the TiN can serve as a better substrate for Ag^0^ loading, which can allow H_2_O_2_ to enter the nanocomposites with rough surface more easily and have more chances to react with the attached Ag^0^.

**Figure 6:** CVs of TiN/SMS (**a**) and Ag-TiN/SMS (**b**) electrodes at the scan rate of 20 mV⋅s^−1^ with addition different concentrations of H_2_O_2_ (0, 0.5, 1.0, 2.0, 3.0, 4.0 mM); (**c**) CVs of Ag-TiN/SMS electrodes in the presence of 2 mM H_2_O_2_ at different the scan rates (20, 40, 60, 80, 100 mV⋅s^−1^); (**d**) The relation of *I*_p_ and ν^1/2^at Ag-TiN/SMS; (**e**) the relation of ln*I*_p_ and (*E*_p_ − *E*_1/2_) at Ag-TiN/SMS.

The electrochemical property of Ag-TiN/SMS electrodes towards H_2_O_2_ reduction was detected by changing the scanning rate. According to Fig. 6c, the reduction peak current increased with the increment of the scan rates in the range of 20–100 mV s^−1^. Besides that, there is a linear relation between the square root of scan rates and the reduction peak currents shown in Fig. 6d, indicating that the process is also probably diffusion controlled, which is perfect for quantitative determination. According to the formula, the diffusion coefficient (D_0_) and reaction rate constant (*k*_0_) are calculated by Eqs. (1), (2)^40^.

1 $$ I_{p} = 2.99 \times 10^{5} n^{3/2} \alpha^{1/2} AC_{0} D_{0}^{1/2} v^{1/2} $$

2 $$ I_{{\text{p}}} = \, 0.{227}n\,F\,A\,C_{0} k_{0} {\text{exp }}[ - aF(E_{{\text{p}}} - E_{{{1}/{2}}} ){/}RT] $$

Figure 6d is the relation of *I*_p_ and *v*^1/2^ at Ag-TiN/SMS, which shows linear section with the linear relationship of *I*_p_ = 84.237*v*^*1/2*^ + 4.060 (R^2^ = 0.996). The calculated *D*_0_ value on Ag-TiN/SMS electrode is 1.69 × 10^–3^ cm s^−1^.

Figure 6e is the relation of ln*I*_p_ and (*E*_p_ − *E*_1/2_) at Ag-TiN/SMS, which shows linear section with the linear relationship of ln*I*_p_ = –11.608 (E_p_ − E_1/2_) − 11.945 (R^2^ = 0.993). The calculated *k*_0_ value on Ag-TiN/SMS electrode is 2.10 × 10^–6^ cm s^−1^.

To better illustrate the relative enhancement of the catalytic activity on Ag-TiN/SMS, electrochemical impedance spectroscopy (EIS) is carried out under the same experimental conditions to investigate the interfacial properties of TiN/SMS and Ag-TiN/SMS electrodes. The obtained Nyquist plots are shown in Fig. 7. The parameters obtained from the fitting curves of EIS are shown in Table 1. The Rp of TiN/SMS and Ag-TiN/SMS electrodes are 571 Ω and 539 Ω, and the Rct of them are113.7 k Ω and30.36 k Ω, respectively. The change can be ascribed to the high conductivity of TiN. Ag-TiN/SMS electrodes provide a good electron pathway between the electrodes and electrolyte and could accelerate the electro transfer rate.

**Figure 7:** Electrochemical impedance Nyquist plots of Ag-TiN/SMS (red filled circle) and TiN/SMS (black filled square) electrodes 0.02 M PBS (pH7.0), Amplitude of 5 mV from 10^–2^ ~ 10^5^ Hz with bias voltage of − 0.4 V.

**Table1:** Parameters obtained from the fitting curves of EIS in Fig. 7.

Samples	*R*_s_ (Ω)	*R*_p_ (Ω)	*R*_ct_ (kΩ)
Ag-TiN/SMS	124.3	539	30.36
TiN/SMS	129.1	571	113.7

### Detection performance of Ag-TiN/SMS towards H_2_O_2_

Amperometric I-t curves were performed with the successive addition H_2_O_2_ into a stirring electrochemical cell containing 3 mL PBS (0.02 M, pH 7.0) at an optimized potential of − 0.3 V (Fig. 8a). The inner diagram in the figure is an enlarged version of the 0–400 s. For Ag-TiN/SMS electrode, each response current step showed a smooth trend between 0.5 and 2100 μM. It means that Ag-TiN/SMS electrode can quickly reach a stable response current over a wide range of concentrations. This may be the stability of the electrode material was improved after nitriding. And the electron transfer rate of the Ag-TiN/SMS is increased during the nitriding process.

**Figure 8:** (**a**) Amperometric responses (I–t) of Ag-TiN/SMS in 0.02 M PBS (pH 7.0) with the successive adding H_2_O_2_; (**b**)The current concentration (I–C) linear fitting results for Ag-TiN/SMS.

Figure 8b shows the linear fitting relationships between the current responses with different concentrations of H_2_O_2_. To regress from the I-t tests results for Ag-TiN/SMS electrodes. Their current responses as functions of H_2_O_2_ concentration can be represented by three different linear equations, which are valid at different concentration ranges. The linear regression equations of Ag-TiN/SMS are I(μA) = 2.351 ${\text{C}}_{{{\text{H}}_{{2}} {\text{O}}_{{2}} }}$ (mM) + 0.444 (R^2^ = 0.989) for ${\text{C}}_{{{\text{H}}_{{2}} {\text{O}}_{{2}} }}$ = 0.05–252 μM, I(μA) = 1.507 ${\text{C}}_{{{\text{H}}_{{2}} {\text{O}}_{{2}} }}$ (mM) + 0.663 (R^2^ = 0.996) for ${\text{C}}_{{{\text{H}}_{{2}} {\text{O}}_{{2}} }}$ = 252–785 μM and I (μA) = 1.067 ${\text{C}}_{{{\text{H}}_{{2}} {\text{O}}_{{2}} }}$ (mM) + 1.012 (R^2^ = 0.999) for ${\text{C}}_{{{\text{H}}_{{2}} {\text{O}}_{{2}} }}$ = 785–2100 μM. The limit of detection (LOD) was determined by using the equation LOD = 3*S*_B_/*b*. Where *b* is the slope of the calibration curve and *S*_B_ is the standard deviation of the blank solution. The LOD (S/N = 3) of Ag-TiN/SMS sensor is calculated to be 7.7 nM. The obtained sensitivity of Ag-TiN/SMS is 33.25 μA mmol L^−1^ cm^−2^. There results demonstrate that Ag-TiN/SMS provides a facile but effective method to fabricate high-performance electrode in sensing applications.

Compare the reports of various hydrogen peroxide sensors, as shown in Table 2, the Ag-TiN/SMS exhibited the lowest detection limit with good linear range and the fast-current response towards H_2_O_2_. Perhaps in the composite, titanium nitride may play an important role as a substrate led to the response time of the Ag-TiN/SMS about hydrogen peroxide was significantly shortened and the electron transfer rate goes up.

**Table2:** Comparison of H_2_O_2_ sensors reported previously with Ag-TiN/SMS sensor.

Sensors	Linear range (μM)	Detection limit (μM)	References
PB-TiO_2_	1.5–90	1.5	^41^
TN/DNA/nano-TiO_2_	50–22,300	50	^42^
TiN	20–3000	250	^30^
AgNPs-TiO_2_ NB/GCE	100–60,000	1.7	^43^
GC/TiNnp/NH_2_-IL	0–2100	0.1	^44^
Cu_2_O/TiO_2_/SEP	20–2360	1.7	^45^
Cu_2_O/TiO_2_/Ti	500–8000	90.5	^46^
Au/TiO_2_	5–100	4	^47^
Co_3_N NW/TM	0.1–2500	0.05	^48^
CdSe@ZnS/AgNCs	0.5–60	0.3	^49^
Ag-TiN/SMS	0.05–2100	0.0077	This work

### Selectivity, long-term stability, reproducibility and repeatability of Ag-TiN/SMS

In the process of electrochemical detection, the interference study is a very important aspect in the determination of any species. To detect selectivity of Ag-TiN/SMS, the modified electrode was evaluated in the presence of common interfering electroactive substances such as vitamin C (VC), uricacid (UA), L-glucose (L-Glu), glycine (Gly) and lactosum (Lac) in PBS. As shown in Fig. 9a, the current responses about 0.5 mM vitamin C, uricacid, L-glucose, glycine and lactosum were negligible when compared with 0.1 mM H_2_O_2_. Thus, Ag-TiN/SMS electrode exhibited highly selectivity for H_2_O_2_ detection.

**Figure 9:** (**a**) Amperometry responses (I–t) of Ag-TiN/SMS electrode in the presence of five different interfering species (0.5 mM VC,0.5 mM UA,0.5 mM L-Glu, 0.5 mM Gly, 0.5 mM Lac); (**b**) Normalized response of Ag-TiN/SMS toward 0.5 mM H_2_O_2_ in PBS (pH 7.0) at − 0.3 V in 30 days; (**c**) reproducibility studies; (**d**) repeatability studies.

The long-term stability of sensor was investigated over a 30-day period (Fig. 9b). The current response to 0.5 mM of H_2_O_2_ maintained about 91.67% of the original value after the storage period of 30 days. It follows that TiN/SMS substrate material can help silver nanoparticles grow uniformly and contribute to the good stability.

To study the sensor reproducibility, eight Ag-TiN/SMS sensors were prepared by the same method and tested for the H_2_O_2_ (0.5 mM) under the same condition (Fig. 9c). The relative standard deviation (RSD) of the response on these eight electrodes is 1.9% by calculation, showing an acceptable reproducibility. Moreover, the RSD of the response repeated for five succeeding measurements is 1.5%. Obviously, the proposed Ag-TiN/SMS electrode demonstrated outstanding repeatability (Fig. 9d).

### Real sample analysis

To investigate the potentials of the sensor to real samples, the Ag-TiN/SMS was evaluated. Different concentrations of H_2_O_2_ solutions were prepared using the diluted milk sample. According to FDA, the concentration of H_2_O_2_ in milk samples should be less than 14.6 μM^40^. Hence, in order to further explore the possible effectivity of the developed sensor to real sample analysis, various concentrations of these solutions were added to the electrochemical cell containing 3 mL PBS and the amperometry responses were recorded. As is listed in Table 3, the recovery was in the range of 97.00–102.01%, suggesting that the proposed sensor can be applied to detection of H_2_O_2_ in practical. The milk sample without H_2_O_2_ did not show any detectable signal.

**Table 3:** Determination of H_2_O_2_ in milk sample solutions.

Sample	C_added_ (μM)	C_founded_ (μM)	Recovery (%)
1	0.1	0.0970	97.00
2	0.5	0.4929	98.58
3	1.0	1.0002	100.02
4	1.5	1.4981	99.87
5	2.0	2.0402	102.01

## Conclusions

In brief, the Ag-TiN/SMS was successfully prepared by one-pot solvothermal reaction and subsequent nitridation, and then directly applied in a non-enzymatic electrochemical determination of H_2_O_2_. The Ag-TiN/SMS exhibited the excellent catalytic activity towards H_2_O_2_. Electrochemical experiment results show that the presence of Ag^0^ and TiN/SMS were both responsible for the greatly enhanced performance of sensor. The fabricated Ag-TiN/SMS electrode shows high reproducibility, great analytical selectivity, sensitivity, and stability, making it one of the promising candidates for efficient and sensitive determination of H_2_O_2_. Furthermore, amperometric characterization revealed that the developed non-enzymatic electrochemical sensor for detection of H_2_O_2_ from 0.05 to 2100 μM was effective, and the detection limit can reach as low as 7.7 nM (S/N = 3). For real samples, the fabricated sensor also reliably applied in detection of H_2_O_2_ at milk.

## Abbreviations

SMS: Submicrospheres
UA: Uric acid
L-Glu: L-glucose
Gly: Glycine
Lac: Lactosum
TBOT: Tetrabutyl titanate
LOD: Limit of detection
RSD: Relative standard deviation
FDA: Food and drug administration

## References

[1] Kalambate PK, Rao Z, Wu J, Shen Y, Boddula R, Huang Y (2020). Electrochemical (bio) sensors go green. Biosens. Bioelectron..

[2] Balasubramanian P, Annalakshmi M, Chen SM, Sathesh T, Peng TK, Balamurugan TST (2018). Facile solvothermal preparation of Mn_2_CuO_4_ microspheres: excellent electrocatalyst for real-time detection of H_2_O_2_ released from live cells. ACS Appl. Mater. Interfaces.

[3] Ma B, Kong C, Hu X, Liu K, Huang Q, Lv J, Lu W, Zhang X, Yang Z, Yang S (2018). A sensitive electrochemical nonenzymatic biosensor for the detection of H_2_O_2_ released from living cells based on ultrathin concave Ag nanosheets. Biosens. Bioelectron..

[4] Asif M, Liu H, Aziz A, Wang H, Wang Z, Ajmal M, Xiao F, Liu H (2017). Core-shell iron oxide-layered double hydroxide: high electrochemical sensing performance of H_2_O_2_ biomarker in live cancer cells with plasma therapeutics. Biosens. Bioelectron..

[5] Bai Z, Li G, Liang J, Su J, Zhang Y, Chen H, Huang Y, Sui W, Zhao Y (2016). Non-enzymatic electrochemical biosensor based on Pt NPs/RGO-CS-Fc nano-hybrids for the detection of hydrogen peroxide in living cells. Biosens. Bioelectron..

[6] Liu ZT, Ye JS, Hsu SY, Lee CL (2018). A sonoelectrochemical preparation of graphene nanosheets with graphene quantum dots for their use as a hydrogen peroxide sensor. Electrochim. Acta.

[7] Sheng YY, Yang HL, Wang Y, Han L, Zhao YJ, Fan A (2017). Silver nanoclusters-catalyzed luminol chemiluminescence for hydrogen peroxide and uric acid detection. Talanta.

[8] Üzer A, Durmazel S, Erçağ E, Apak R (2017). Determination of hydrogen peroxide and triacetone triperoxide (TATP) with a silver nanoparticles—based turn-on colorimetric sensor. Sens. Actuators B Chem..

[9] Wang LZ, Liu Y, Yang ZP, Wang YY, Rao HB, Yue GZ, Wu CM, Lu CF, Wang XX (2020). A ratiometric fluorescence and colorimetric dual-mode assay for H_2_O_2_ and xanthine based on Fe, N co-doped carbon dots. Dyes Pigment..

[10] Li H, Zhao HL, He HY, Shi LB, Cai X, Lan MB (2018). Pt-Pd bimetallic nanocoral modified carbon fiber microelectrode as a sensitive hydrogen peroxide sensor for cellular detection. Sens. Actuators B Chem..

[11] Liu J, Bo XJ, Yang J, Yin DD, Guo LP (2017). One-step synthesis of porphyrinic iron-based metal-organic framework/ordered mesoporous carbon for electrochemical detection of hydrogen peroxide in living cells. Sens. Actuators B Chem..

[12] Asif M, Wang HT, Dong S, Aziz A, Zhang G, Fei X, Liu HF (2017). Metal oxide intercalated layered double hydroxide nanosphere: with enhanced electrocatalyic activity towards H_2_O_2_ for biological applications. Sens. Actuators B Chem..

[13] Dai H, Chen Y, Niu X, Pan C, Chen H, Chen X (2018). High-performance electrochemical biosensor for nonenzymatic H_2_O_2_ sensing based on Au@C-Co_3_O_4_ heterostructures. Biosens. Bioelectron..

[14] Guler M, Turkoglu V, Bulut A, Zahmakiran M (2018). Electrochemical sensing of hydrogen peroxide using Pd@Ag bimetallic nanoparticles decorated functionalized reduced graphene oxide. Electrochim. Acta.

[15] Antink WH, Choi Y, Seong K, Piao Y (2018). Simple synthesis of CuO/Ag nanocomposite electrode using precursor ink for non-enzymatic electrochemical hydrogen peroxide sensing. Sens. Actuators B Chem..

[16] Tian LL, Xia KD, Hu WP, Zhong XH, Chen YL, Yang C, He GG, Su YY, Li L (2017). A wide linear range and stable H_2_O_2_ electrochemical sensor based on Ag decorated hierarchical Sn_3_O_4_. Electrochim. Acta.

[17] Chou YJ, Ningsih HS, Shih SJ (2020). Preparation, characterization and investigation of antibacterial silver-zinc co-doped β-tricalcium phosphate by spray pyrolysis. Ceram. Int..

[18] Nawaz T, Sengupta S, Yang CL (2019). Silver recovery as Ag(0) nanoparticles from ion-exchange regenerant solution using electrolysis. J. Environ. Sci. (China).

[19] Manno R, Sebastian V, Irusta S, Mallada R, Santamaria J (2020). Ultra-small silver nanoparticles immobilized in mesoporous SBA-15. Microwave-assisted synthesis and catalytic activity in the 4-nitrophenol reduction. Catal. Today..

[20] Lengv ZY, Wu DR, Yang QK, Zeng SC, Xia WS (2018). Facile and one-step liquid phase synthesis of uniform silver nanoparticles reduction by ethylene glycol. Optik.

[21] Lorestani F, Shahnavaz Z, Mn P, Alias Y, Manan NSA (2015). One-step hydrothermal green synthesis of silver nanoparticle-carbon nanotube reduced-graphene oxide composite and its application as hydrogen peroxide sensor. Sens. Actuators B Chem..

[22] Wu F, Lin Q, Wang L, Zou Y, Chen M, Xia Y, Lan J, Chen J (2020). A DNA electrochemical biosensor based on triplex DNA-templated Ag/Pt nanoclusters for the detection of single-nucleotide variant. Talanta.

[23] Lin CY, Lai YH, Balamurugan A, Vittal R, Lin CW, Ho KC (2010). Electrode modified with a composite film of ZnO nanorods and Ag nanoparticles as a sensor for hydrogen peroxide. Talanta.

[24] Do JY, Kim J, Jang Y, Baek YK, Kang M (2018). Change of band-gap position of MTiO_2_ particle doped with 3d-transition metal and control of product selectivity on carbon dioxide photoreduction. Korean J. Chem. Eng..

[25] Paola AD, Bellardita M, Palmisano L (2013). Brookite, the least known TiO_2_ photocatalyst. Catalysts.

[26] Yamamoto T, Wada Y, Yin H, Sakata T, Mori H, Yanagida S (2002). Microwave-driven polyol method for preparation of TiO_2_. Nanocrystallites.

[27] Ren M, Xu H, Li F, Liu WL, Gao CL, Su LW, Li GD, Hei JP (2017). Sugarapple-like N-doped TiO_2_ @carbon core-shell spheres as high-rate and long-life anode materials for lithium-ion batteries. J. Power Sources.

[28] Yan D, Yu CY, Zhang XJ, Li JB, Li JF, Lu T, Pan LK (2017). Enhanced electrochemical performances of anatase TiO_2_ nanotubes by synergetic doping of Ni and N for sodium-ion batteries. Electrochim. Acta.

[29] Chen P, Li HP, Hu SY, Zhou T, Yan YW, Pan W (2015). Copper-coated TiN nanofibers with high electrical conductivity: a new advance in conductive one-dimensional nanostructures. J. Mater. Chem. C.

[30] Xie Z, Liu XX, Wang WP, Liu C, Li ZC, Zhang ZJ (2014). Fabrication of TiN nanostructure as a hydrogen peroxide sensor by oblique angle deposition. Nanoscale Res. Lett..

[31] Skovager A, Whitehead K, Wickens D, Verran J, Ingmer H, Arneborg N (2013). A comparative study of fine polished stainless steel, TiN and TiN/Ag surfaces: adhesion and attachment strength of Listeria monocytogenes as well as anti-listerial effect. Colloids Surf. B Biointerfaces.

[32] Dong S, Chen X, Gu L, Zhang L, Zhou X, Liu Z, Han P, Xu H, Yao J, Zhang X, Li L, Shang C, Cui G (2011). A biocompatible titanium nitride nanorods derived nanostructured electrode for biosensing and bioelectrochemical energy conversion. Biosens. Bioelectron..

[33] Xiao YH, Zhan GH, Fu ZG, Pan ZC, Xiao CM, Wu SK, Chen C, Hu GH, Wei ZG (2014). Robust non-carbon titanium nitride nanotubes supported Pt catalyst with enhanced catalytic activity and durability for methanol oxidation reaction. Electrochim. Acta.

[34] Wang Y, Yuan HY, Lu XL, Zhou ZD, Xiao D (2006). All solid-state pH electrode based on titanium nitride sensitive film. Electroanalysis.

[35] Saadati S, Salimia A, Hallaj R, Rostami A (2014). Direct electron transfer and electrocatalytic properties of immobilized hemoglobin onto glassy carbon electrode modified with ionic-liquid/titanium-nitride nanoparticles: application to nitrite detection. Sens. Actuators B Chem..

[36] Xie YB, Xia C, Du HX, Wang W (2015). Enhanced electrochemical performance of polyaniline/carbon/titanium nitride nanowire array for flexible supercapacitor. J. Power Sources.

[37] Lee JH, Lim JY, Lee CS, Park JT, Kim JH (2017). Direct growth of NiO nanosheets on mesoporous TiN film for energy storage devices. Appl. Surf. Sci..

[38] Chen Y, Deng Y, Pu Y (2016). One pot preparation of silver nanoparticles decorated TiO_2_ mesoporous microspheres with enhanced antibacterial activity. Mater. Sci. Eng..

[39] Zhao FM, Wen G, Kong LY (2017). Electrochemical performance of titanium nitride nanotubes as negative electrode in a static vanadium battery towards V(II)/V(III) redox couple. Chin. J. Inorg. Chem..

[40] Bard AJ, Faulkner LR (2001). Electrochemical Methods Fundamentals and Applications.

[41] Chu ZY, Shi L, Liu Y, Jin WQ, Xu NP (2013). In-situ growth of micro-cubic Prussian blue–TiO_2_ composite film as a highly sensitive H_2_O_2_ sensor by aerosol co-deposition approach. Boisens. Bioelectron..

[42] Lo PH, Kumar SA, Chen SM (2008). Amperometric determination of H_2_O_2_ at nano-TiO_2_/DNA/thionin nanocomposite modified electrode. Colloids Surf. B.

[43] Qin X, Lu W, Luo Y, Chang G, Asiri AM, Al-Youbi AO, Sun X (2012). Green photocatalytic synthesis of Ag nanoparticle-decorated TiO_2_ nanowires for nonenzymaticamperometric H_2_O_2_ detection. Electrochim. Acta.

[44] Saadati S, Salimi A, Hallaj R, Rostami A (2012). Layer by layer assembly of catalase and amine-terminated ionic liquid onto titanium nitride nanoparticles modified glassy carbon electrode: study of direct voltammetry and bioelectrocatalytic activity. Anal. Chim. Acta.

[45] Yan P, Zhong LF, Wen X (2018). Fabrication of Cu_2_O/TiO_2_/sepiolite electrode for effectively detecting of H_2_O_2_. J. Electroanal. Chem..

[46] Wen X, Long M, Tang AD (2017). Flake-like Cu_2_O on TiO_2_ nanotubes array as an efficient nonenzymatic H_2_O_2_ biosensor. J. Electroanal. Chem..

[47] Peng XG, Wan GP, Wu LH (2018). Peroxidase-like activity of Au@TiO_2_ yolk-shell nanostructure and its application for colorimetric detection of H_2_O_2_ and glucose. Sens. Actuators B.

[48] Xie FY, Cao XQ, Qu FL, Asiri AM, Sun XP (2018). Cobalt nitride nanowire array as an efficient electrochemical sensor for glucose and H_2_O_2_ detection. Sens. Actuators B Chem..

[49] Zhou Z, Yang L, Huang L, Liao Y, Liu Y, Xiao Q (2020). A novel fluorescent probe for H2O2 detection based on CdSe@ZnS quantum dots/Ag nanocluster hybrid. Anal. Chim. Acta.

